The article "Diagnostic value for methylation in cervical cancer based on a small‐molecule fluorescent probe targeting DNMT1" was retracted in 2025. Reasons: duplicate publication; overlap with earlier publications; compromised peer review; a compromised editor.

# Diagnostic value for methylation in cervical cancer based on a small‐molecule fluorescent probe targeting DNMT1

**DOI:** 10.1111/srt.70042

**Published:** 2024-09-04

**Authors:** Baohua Yang, Chao Xu, Hang Li, Xiuxiang Zhu, Ziyin Xia, Ling Xu, Qian Zhang

**Affiliations:** ^1^ Department of Obstetrics and Gynecology Minhang Hospital Fudan University Shanghai China; ^2^ Department of Medicinal Chemistry School of Pharmacy Fudan University Shanghai China

**Keywords:** cervical cancer, diagnostic value, fluorescent probe, genetic testing technology, methylation, small‐molecule

## Abstract

**Background:**

Value analysis of a small‐molecule fluorescent probe for methylation detection in different cervical lesions.

**Materials and Methods:**

(1) The grayscale values of distinct lesion tissues were remarkably distinct among the four groups (*p* < 0.05). The comparison of the grayscale value between the two groups showed that the CA group noticeably exceeded the LSIL and cervicitis groups, and the HSIL group was apparently higher than the LSIL and cervicitis groups (*p* < 0.05); (2) The mean grayscale values of the enrolled subjects were calculated with 55.21 as the midline, with >55.21 as positive and ≤55.21 as negative.

**Results:**

The results showed that the positive rate of the cervicitis group was 0.00%, the LSIL group 67.74%, the HSIL group 83.33%, and the CA group 100.00%. The results among the four groups were notably distinct (*p <* 0.05); (3) The comparison among DAPI, probe, bright, and merged images of cervicitis, LSIL, HSIL, and CA indicated that different cervical lesions were with quite various stains.

**Conclusion:**

The grayscale value, positive rate, and stained picture of distinct cervical lesions were remarkably different. The small‐molecule fluorescent probe has a good value in differentiating cervical lesions and can be considered for popularization and application.

## 1 INTRODUCTION

Cervical cancer is the most common gynecological malignant tumor, which poses a serious threat to women's health.^1^ The number of new cases of cervical cancer worldwide in 2020 was 604 127; The death case is 341 831. the number of new cases in Asia is accounting for about 50% of the world's total. At present, the number of cases of cervical cancer is as high as 30 000 per year, which has become a worldwide public health problem.^2^, ^3^

Screening methods used in cervical cancer most widely are cervical liquid‐based cytology and high‐risk HPV detection, but both of the above methods have some limitations.^4^, ^5^ For example, liquid‐based cytology has low sensitivity, uneven sampling, slide preparation, and reading levels of cytological pictures, lack of standardized quality control, and strong subjective dependence.^6^ Although high‐risk HPV detection is highly sensitive, transient HPV infection and pathogenic persistent infection cannot be distinguished, while women of reproductive age have a higher HPV infection rate, suggesting that HPV screening alone is of weak significance.^7^, ^8^ The application of molecular biology detection in the screening of cervical cancer has been popularized.

The article "Diagnostic value for methylation in cervical cancer based on a small‐molecule fluorescent probe targeting DNMT1" was retracted in 2025. Reasons: duplicate publication; overlap with earlier publications; compromised peer review; a compromised editor.

## 2 MATERIALS AND METHODS

### 2.1 General data

Cervical tissues from 81 patients who visited our cervical specialist clinic from August 2020 to January 2022 were retrospectively registered, and the enrolled tissues were divided into cervicitis group (*n = *23), LSIL (*n = *31), HSIL (*n = *18), and CA (*n = *9) based on histopathological diagnosis as the gold standard.

Inclusion criteria: (1) Clinical medical records were complete; (2) pathological examination was performed in our hospital; (3) application was approved by the Ethics Association of the hospital.

Exclusion criteria: (1) Patients with other malignant tumors; (2) patients with mental illness; (3) participating in other ongoing clinical research; (4) drug or alcohol dependents.

### 2.2 Quantitative detection of DNMT1 by a small‐molecule fluorescent probe in cervical cell

PAX1 methylation is primarily mediated by DNA methyltransferase 1 (DNMT1), and DNMT1 plays an important role as a PAX1 methylation promoter in cervical cancer cells. Our team, in collaboration with the Pharmaceutical Chemistry Laboratory of Fudan University, designed and synthesized a small fluorescent probe RG108‐FITC (patent number: CN201910750081.X), deriving from the combination of ligands or inhibitors of DNMT1 with the specific fluorescent group. DNMT1 level in cells can be measured via the probe by specifically binding to DNMT1, so indirectly evaluating the methylation level of PAX1. For quantitative DNMT1 fluorescence assays, the cells were diluted with medium, counted, and transferred to a new centrifuge tube after centrifuging the cell suspension, and then an appropriate volume of medium containing the small‐molecule fluorescent probe was added until the volume was up to 1 mL. After incubation at 37°C for 4 h, the cells were harvested and treated with DAPI (0.1 µg/mL) for 10 min to stain cell nuclei. Images of DAPI and fluorescent probes were obtained by confocal fluorescence microscopy (Nikon) at 349 and 488 nm, respectively. Fluorescence intensity was calculated by ImageJ.

### 2.3 Outcome measurements

The primary outcome was the efficacy of the probe in differentiating various cervical lesions in terms of methylation. The grayscale values of distinct cervical lesions were detected and contrasted. Meanwhile, the mean grayscale values of enrolled tissues (55.21) were set as the cut‐off point to evaluate the positive rate, and the comparison between groups was carried out. Finally, the stained pictures of typical cases in the cervicitis, LSIL, HSIL, and CA groups were screened for comparison.

The article "Diagnostic value for methylation in cervical cancer based on a small‐molecule fluorescent probe targeting DNMT1" was retracted in 2025. Reasons: duplicate publication; overlap with earlier publications; compromised peer review; a compromised editor.

### 2.4 Statistical methods

The results were expressed as mean ± standard deviation. Data that did not conform to a normal distribution were statistically calculated using the Kruskal Wallis rank sum test, and the results were expressed as median and quartiles. Enumeration data were expressed as rates, and statistics were performed by chi‐square test. Differences were considered significant at *p *< 0.05. GraphPad Prism 8.3 was conducted for plotting.

## 3 RESULTS

### 3.1 Comparison of the greyscale values of the small‐molecule probe in distinct cervical lesion cell

A comparison of the greyscale values of the small‐molecule probe in distinct lesion tissues suggested that the difference was remarkable among all groups (*p *< 0.001). Comparison between the two groups revealed that the greyscale value in the CA group was noticeably higher than that in the LSIL and cervicitis groups (*p *< 0.05), and in the HSIL group, the greyscale values considerably exceeded that of the LSIL and cervicitis groups (*p *< 0.05). Table 1 shows a comparison of small‐molecule probe greyscale values for distinct cervical lesion tissues, Figure 1 shows a comparison of the greyscale values of the small‐molecule probe in distinct cervical lesion tissues.

**TABLE 1:** Comparison of small‐molecule probe greyscale values for distinct cervical lesion tissues ($\bar{x}\pm s$).

Group	Cases	Grayscale values
Cervicitis group	23	24.88 ± 13.39
LSIL	31	61.30 ± 23.18
HSIL	18	71.62 ± 12.60^a,b^
CA	9	78.91 ± 8.22^a,b^
*t*		34.477
*p*	–	<0.001

^a,b^ Represent *p *< 0.05, contrasted to the cervicitis and the LSIL group, respectively.

**FIGURE 1:** Comparison of the greyscale values of the small‐molecule probe in distinct cervical lesion tissues. The greyscale values were strikingly higher in the CA group in contrast to the LSIL and cervicitis groups, and the HSIL group was found a notable increase compared with the LSIL and cervicitis groups (both *p *< 0.05).

### 3.2 Evaluate the positive rate of the grayscale values in distinct lesion tissues

Taking the mean grayscale value of 55.21 as the midline, >55.21 as the positive, and ≤55.21 as the negative, the positive rates of the grayscale values of distinct lesion tissues were calculated, respectively. The results suggested that the positive rate of the cervicitis group was 0.00%, the LSIL group 67.74%, the HSIL group 83.33%, and the CA group 100.00%. The positive rate among the four groups was strikingly distinct (*p <* 0.05). Further pairwise comparison indicated that the positive rate of the CA group was superior to that of the cervicitis group, LSIL, and HSIL group, the HSIL group higher than the cervicitis group, and the LSIL group higher than the cervicitis group (all *p <* 0.05), Table 2 shows positive rate of the greyscale values in distinct cervical lesions. Figure 2 shows the difference in the greyscale values of distinct lesions.

The article "Diagnostic value for methylation in cervical cancer based on a small‐molecule fluorescent probe targeting DNMT1" was retracted in 2025. Reasons: duplicate publication; overlap with earlier publications; compromised peer review; a compromised editor.

**TABLE 2:** Positive rate of the greyscale values in distinct cervical lesions.

Group	Cases	Number of greyscale‐positive cases	Positive rate
Cervicitis Group	23	0	0.00%
LSIL	31	21	67.74%^a^
HSIL	18	15	83.33%^a^
CA	9	9	100.00%^a,b,c^
*t*	–	–	6.321
*p*	–	–	<0.001

^a,b,c^ Represent *p* < 0.05, contrasted to the cervicitis, the LSIL, and the HSIL group, respectively.

**FIGURE 2:** Difference in the greyscale values of distinct lesions. The positive rates of the greyscale in distinct cervical tissues were significantly different (*p *< 0.05). Further two‐by‐two comparison showed that the positive rate in the CA group was higher than that in the cervicitis, LSIL, and HSIL, the HSIL group higher than the cervicitis group, and the LSIL group higher than the cervicitis group (*p *< 0.05).

### 3.3 Stained images of typical cases

With DAPI images, probe images, bright images, and merged images of patients with cervicitis, LSIL, HSIL, and CA screened for Comparison, it is more evident that the stained images of patients with distinct cervical lesions varied greatly. Figure 3 shows stained images of patients with cervicitis, and Figure 4 shows stained images of patients with LSIL. Figure 5 shows Stained images of patients with HSIL; Figure 6 shows stained images of patients with cervical cancer.

**FIGURE 3:** Stained images of patients with cervicitis. (A) DAPI image, (B) probe image, (C) bright image, and (D) merged image.

**FIGURE 4:** Stained images of patients with LSIL. (A) DAPI image, (B) probe image, (C) bright image, and (D) merged image.

**FIGURE 5:** Stained images of patients with HSIL. (A) DAPI image, (B) probe image, (C) bright image, and (D) merged image.

**FIGURE 6:** Stained images of patients with cervical cancer. (A) DAPI image, (B) probe image, (C) bright image, and (D) merged image.

## 4 DISCUSSION

In recent years, some areas have shown an obvious tendency to rejuvenation for cervical cancer, with an average age of 52 years of carcinoma onset in situ having subsided to 30–34 years, nearly 20 years earlier than invasive cancer.^9^, ^10^ In China, the age of onset of cervical cancer has also gradually decreased in recent years.^11^, ^12^ 130 000 new cases, and 53 000 deaths due to cervical cancer in China each year, accounting for about 18% of cervical cancer deaths worldwide.^13^, ^14^

Methylation is a type of chemical modification of DNA, which refers to the process by which methyltransferases covalently bind the methyl group of S‐adenosylmethionine to the cytosine 5′ carbon of CpG dinucleotides in the DNA sequence without changing the DNA sequence. Methylation modification of cytosine in DNA plays a crucial role in gene regulation to cell growth and development.^15^, ^16^ Methylation is not only a vital element in maintaining normal biological functions, but is closely related to the occurrence and development of many diseases, such as extensive hypomethylation in tumors, massive demethylation of retrotransposons, and hypermethylation of specific CpG islands. It can be said that aberrant methylation of DNA is an early phase in the process of tumorigenesis, and early screening for methylated genes will help provide new ideas for the diagnosis and healing of tumors.^17^, ^18^

Gene epigenetic modification is the main feature of cervical cancer, and a large number of genes such as shooting cell cycle regulation, apoptosis, DNA repair, and WNT pathway have been confirmed to have methylation modification phenomena, and studies have shown that the activity of DNA de novo methylase DNMTs is directly increased in patients with high‐risk HPV infection, which confirms the correlation between methylation and the pathological process of cervical cancer.^19^, ^20^, ^21^ In the present paper, 81 patients with distinct cervical lesions were examined by a gene detection technique via a small‐molecule fluorescent probe to explore the application value of this method in distinguishing different cervical lesion types. The results showed that there were remarkable differences in the cervicitis, LSIL, HSIL, and cervical cancer patients in terms of quantitative data of the grayscale values. Further comparison of the positive rates according to the mean values showed that there were also noticeable differences among distinct cervical lesion tissues, and the pairwise comparison also had certain statistical significance.

The article "Diagnostic value for methylation in cervical cancer based on a small‐molecule fluorescent probe targeting DNMT1" was retracted in 2025. Reasons: duplicate publication; overlap with earlier publications; compromised peer review; a compromised editor.

Previous in vitro experiments have confirmed that the degree of methylation is associated with the degree of cervical lesions and the course of high‐grade endocervical neoplasia during carcinogenesis. Although there are differences in the methylation time of different genes, the methylation level will increase with the process of carcinogenesis overall which is correlated with the severity of cervical diseases. Therefore, the methylation status of genes can be used as an evaluation of the degree of cervical lesions.^22^, ^23^ A comparison of stained images proved that a significant variety existed in distinct cervical lesions. Although the judgment of stained degree was affected by individual subjective consciousness and detection instruments, the result also confirmed that the methylation level was closely related to the extent of cervical lesions.

The study demonstrated that the innovation of a small‐molecule fluorescent probe based on gene methylation detection was of high application value in terms of quantitative, qualitative, and picture visualization. The limitation was that the samples came from a single and concentrated source, which may impact the results to a certain extent.

## 5 CONCLUSION

The grayscale value, positive rate, and stained picture of distinct cervical lesions were remarkably distinct. The small‐molecule fluorescent probe based on gene detection technology owned a promising prospect in the identification of cervical lesions and could be considered for popularization and application.

## CONFLICT OF INTEREST STATEMENT

The authors declare no conflicts of interest.

## Data Availability

The data supporting the results of this study are available from the corresponding author.
